# NT-proBNP level as a substitute for myocardial perfusion scan in preoperative cardiovascular risk assessment in noncardiac surgery

**DOI:** 10.1186/s12871-023-02205-x

**Published:** 2023-07-20

**Authors:** Saeede Esmati, Anahita Tavoosi, Saghar Mehrban, Vahideh Laleh Far, Ali Mehrakizadeh, Shayan Shahi, Farnoosh Larti

**Affiliations:** Department of Cardiology, Imam Khomeini Hospital Complex, Tehran University of Medical Sciences, Keshavarz Boulevard, Tehran, 1419733141 Iran

**Keywords:** NT-proBNP, Myocardial perfusion scan, Preoperative cardiovascular risk assessment, Noncardiac surgery

## Abstract

**Background:**

Preoperative cardiovascular risk assessment is one of the main principles before noncardiac surgeries. Cardiac stress imaging, such as myocardial perfusion scan (MPS), is a proposed cardiovascular risk evaluation method according to the latest guidelines. Yet, its efficacy, along with the cost-effectiveness of the method, has been questioned in previous studies. Our study aims to evaluate the utility of N-terminal pro-b-type natriuretic peptide (NT-proBNP) level measurement in predicting postoperative cardiovascular complications in candidates who have undergone an MPS before surgery and compare the results.

**Methods:**

A cohort of 80 patients with a revised cardiac risk index score of one or more who were scheduled for moderate to high-risk noncardiac surgeries and met the criteria to undergo an MPS for risk assessment were included in the study. All of them underwent an MPS one week before surgery. Their preoperative NT-proBNP, troponin levels, and electrocardiograms were obtained one day before surgery and again on day three postoperative. The predictive efficacy of NT-proBNP levels and MPS were compared.

**Results:**

Seventy-eight patients underwent surgery, three of which exhibited a rise in troponin level, six showed changes on electrocardiogram, and pulmonary edema was detected in one, three days after surgery. There was no mortality in our patients. The sensitivity and specificity of the MPS for predicting postoperative cardiovascular complications were 100% and 66%, respectively. MPS also had a positive predictive value of 20% and a negative predictive value of 100% in our study. A 332.5 pg/ml cut-off value for NT-proBNP level yielded a sensitivity of 100%, specificity of 79.2%, positive predictive value of 40%, and negative predictive value of 100%.

**Conclusions:**

Our study reveals the incremental specificity and positive predictive value of NT-proBNP level measurement in preoperative cardiovascular risk evaluation compared to MPS. Given the low feasibility, high costs, and disappointing predictive value of MPS, preoperative NT-proBNP level assessment can be substituted. This method can assist anesthesiologists and surgeons with precisely detecting at-risk patients resulting in taking proper measures to reduce the morbidity and mortality of the proposed patients before and during surgeries.

## Introduction

Annually about 200 million adult individuals undergo major noncardiac surgeries (NCS) worldwide. According to the 2019 global burden of postoperative death, postoperative death has been ranked as the third leading cause of death globally [1]. In a prospective cohort in 2019 conducted on 40,004 individuals who underwent NCS, the overall 30-day mortality rate was 1.8%, and postoperative myocardial injury was reported to be the second most prevalent cause of mortality [2]. Needless to say, patients with cardiovascular risk factors and underlying related diseases are more prone to the mentioned postoperative complications [3].

Preoperative cardiovascular risk assessment is frequently performed using the Revised Cardiac Risk Index (RCRI), first developed in 1999 [4]. Despite its ease of application and accuracy in discriminating between low and high-risk patients regarding cardiovascular events, RCRI does not perform well in predicting all-cause mortality [5]. Therefore, the newest preoperative cardiovascular risk assessment guidelines recommend empowering RCRI by recruiting other assessment tools, such as cardiac biomarkers and stress imaging, and adding them to the existing criteria [6].

According to 2022 European Society of Cardiology (ESC) guidelines, utilization of stress imaging modalities such as myocardial perfusion scan (MPS) is a class I recommendation in patients scheduled for high-risk NCS with poor functional capacity and high clinical risk or likelihood of coronary artery disease (CAD), and a class IIb recommendation for patients undergoing medium-risk surgeries, when ischemia is of concern in those with clinical risk factors and poor functional capacity [6]. Although MPS adds an incremental prognostic value to preoperative risk assessment tools, especially in populations with a high risk of CAD [7], it offers a relatively low positive predictive value (4%) for predicting the risk of postoperative cardiovascular complications and is not cost-effective in specific settings [8]. In this paper, we aim to investigate the difference between the predictive value of preoperative NT-proBNP testing, a frequent biomarker checked in NCS preoperative risk assessment, and MPS, as a stress imaging, in a cohort of patients undergoing moderate to high-risk NCS for predicting postoperative cardiovascular complications.

## Materials and methods

### Study population

A prospective cohort study was performed at Imam Khomeini Hospital, a tertiary referral center in Tehran, Iran. The Tehran University of Medical Sciences ethics committee approved the research protocol under code 41363. Patients were provided detailed information on the research, and their written informed consent was obtained. We conducted a prospective cohort on consecutive patients from October 2018 to February 2020 who were scheduled for elective noncardiac surgeries in the following two weeks and were referred to the cardiology clinic for preoperative cardiovascular risk assessment. Patients exhibiting poor functional capacity (FC) who were scheduled for moderate or high-risk noncardiac surgeries and at least one point of Revised Cardiac Risk Index (RCRI) score in the preoperative evaluation were included. Emergent surgeries or patients undergoing vascular surgeries with an RCRI score < one or patients not meeting the criteria for poor functional capacity were excluded.

### Data collection

While being visited for preoperative assessment, a thorough patient history was taken, and a physical examination was performed. The candidates for elective noncardiac surgery, including abdominal, thoracic, orthopedic, gynecological, neurosurgery, Ear, Nose, and Throat (ENT), and plastic or urological surgeries, were included. All our patients underwent moderate or high-risk surgeries with a risk of intraoperative bleeding, hemodynamic shift, or long operation time. The mentioned plastic surgeries were abdominoplasty and body contouring, which encompass a high risk of intraoperative bleeding and long operation time. The RCRI score for each patient was calculated as follows [4]: one point for each of the six independent factors, including the high-risk type of surgery, ischemic heart disease (IHD), history of congestive heart failure (CHD), history of cerebrovascular disease, insulin therapy for diabetes, and preoperative serum creatinine more than 2.0 mg/dl. Poor FC was defined as the inability to climb two or more flights of stairs or run a short distance based on the patient's history [9].

The study population consisted of patients scheduled for moderate or high-risk noncardiac surgery with poor functional capacity, in whom the RCRI score was >  = one. All patients underwent myocardial perfusion imaging (MPS) within the week before surgery. The patients were divided into four groups based on their MPS results: normal, mild ischemia, moderate ischemia, and severe ischemia. Patients with moderate or severe ischemia in the MPS test or those with RCRI scores > two who had mild ischemia in the MPS test underwent coronary angiography (CAG). In case of subsequent coronary artery bypass graft (CABG) or percutaneous coronary intervention (PCI), their surgery was postponed for six months afterward if possible.

Baseline NT-proBNP, troponin levels, and electrocardiogram (ECG) were obtained one day before surgery. As the patients needed in-hospital blood sampling before surgery, we combined checking NTproBNP with routine lab test sampling for the patient’s convenience preventing double puncture. Patients should be clinically stable in the period of MPS and NT-proBNP measurement. ECG and troponin levels were re-evaluated on the third post-operation day. During post-operation hospitalization, patients were visited daily, and possible cardiovascular complications were investigated. Postoperative cardiovascular complications were considered as one or more of the following:

1. Troponin > 1.0 ng/mL or rising five times higher than upper reference limit for troponin [10] (The CTnI test was performed by an IMMULITE® 2000 XPi system, Siemens device. This test kit had an analytical sensitivity of 0.2ng/mL, and the expected normal values were below 1.0 ng/ml.)
2. ECG changes (new ST-depression, T wave inversion, or pathologic Q-wave)
3. Acute decompensated heart failure (based on physical examination and dramatic response to acute decompensated heart failure treatment)
4. Cardiovascular mortality occurring within 30 days of operation is defined as death due to MI, ventricular fibrillation, complete heart block, or sudden death with no apparent and explainable cause.

It is worth noting that although ECG changes are not equivalent to myocardial injury/infarction, in a postoperative setting where patients receive analgesic medicine, ECG changes or troponin rise might be the only clues to detect a myocardial injury/infarction without symptoms of chest pain or discomfort.

### Statistical analysis

Numerical variables were tested regarding their distribution. Variables with normal distribution were described using median and standard deviation (SD), and median and first and third quartiles (Q1 and Q3) were used to define variables with skewed distribution. Patients with and without postoperative cardiovascular complications were compared using Mann–Whitney U-test for nonparametric continuous variables and Fisher's exact test for categorical variables, where appropriate. A univariate logistic regression model was used to evaluate how well the predictors, including NT-proBNP and MPS, predicted the occurrence of postoperative cardiovascular complications. The receiver operating characteristic (ROC) curve was computed, and the area under the curve (AUC) and its 95% confidence interval (CI) were used to determine the discriminative ability of the predictors. Statistical significance was defined when the p-value was less than 0.05. All the analyses were performed with IBM SPSS version 26.

## Results

### Preoperative assessment

Eighty consecutive patients were selected according to the inclusion and exclusion criteria and were entered into this study. The mean age of the participants was 61.3 years (SD = 10.5), and 55% were men (*n* = 44). Most of our patients had an RCRI score of 2 (*n* = 57, 71.2%), followed by an RCRI score of 3 in 21 (26.3%). RCRI scores of 1 and 4 each accounted for 1.2% of the participants (one patient each). All patients underwent MPS, and the results were as follows: Forty-eight patients (60%) exhibited no sign of ischemia on MPS, whereas mild, moderate, or severe ischemia was detected in 15, 12, and 5 patients respectively (18.8%, 15%, and 6.3% of the study group respectively).

According to the proposed criteria, 26 patients underwent CAG, three (11.5%) of whom were diagnosed with single vessel disease (SVD). Two vessel disease (2VD) and multiple vessel disease (MVD) were detected in 2 (7.6%) and 4 (15.3%) patients, respectively. Of these nine patients, one proceeded to CABG, and one was selected for PCI, so their surgery was postponed for six months. The remaining seven patients with documented coronary artery disease proceeded to their scheduled surgeries with optimized medical treatment (Fig. 1). None of the patients tested positive for troponin before surgery, and their preoperative ECG findings were normal. The median level of NT-proBNP was 148.5 pg/ml before surgery (Q1 = 100, Q3 = 367).

**Fig. 1:** Summary of the study population. All patients underwent MPS. According to the results of MPS and the proposed criteria in the text, CAG was performed on 26 patients. Based on the results of CAG, two patients, who both had moderate ischemia on MPS, were excluded from the study as they turned out to be PCI or CABG candidates, and their NCS surgeries were postponed for six months

### Postoperative assessment

On the third postoperative day, a troponin level of more than 1.0 ng/ml was detected in 3 patients (3.9%). ECG findings revealed ST depression in one patient and T inversion and pathologic Q wave in 3 and 2 patients, respectively. One patient developed pulmonary edema during hospitalization due to acute decompensated heart failure, confirmed by echocardiography, and was treated accordingly. No cases of cardiovascular mortality occurred during the 30-day postoperative period. Overall, postoperative cardiovascular complications were seen in 6 out of 78 patients (7.7%).

Postoperative cardiovascular complications occurred more prevalently among patients with signs of ischemia in the MPS (*p* = 0.002). The sensitivity and specificity of the MPS for predicting postoperative cardiovascular complications were 100% and 66%, respectively. In our study, MPS also had a positive predictive value (PPV) of 20% and a negative predictive value (NPV) of 100%. The detailed data on patient outcomes according to the result of the MPS is summarized in Table 1.

**Table 1:** Efficacy of MPS in predicting postoperative cardiovascular complications

Post Operation Evaluation	MPS findings n (%)				
	Normal	Mild ischemia	Moderate ischemia	Severe ischemia	*p*-value
Positive Troponin	0	0	1 (1.3%)	2 (2.5%)	< 0.001
Pulmonary Edema	0	0	0	1 (1.3%)	-
ECG Findings					
Normal	48 (61.5%)	15 (19.2%)	6 (7.7%)	3 (3.8%)	0.002
ST changes	0	0	0	1 (1.3%)	
T inversion	0	0	2 (2.5%)	1 (1.3%)	
Pathologic Q wave	0	0	2 (2.5%)	0	
Overall CV complications	0	0	4 (5.1%)	2 (2.5%)	0.002

The median level of preoperative NT-proBNP in patients with postoperative cardiovascular complications was 514 pg/ml (Q1 = 411.75, Q3 = 725.5), which was significantly higher than the NT-proBNP in those without postoperative cardiovascular complications (134.5 pg/ml, Q1 = 96.25, Q3 = 288.25, *p* < 0.001, Fig. 2).

**Fig. 2:** Box plot of preoperative NT-proBNP in patients who sustained postoperative cardiovascular complications (*n* = 6) and those who did not (*n* = 72)

The detailed data on patient outcomes regarding the median value of NT-proBNP is summarized in Table 2.

**Table 2:** Summary of NT-proBNP level concerning different postoperative cardiovascular complications

Post operation Evaluation	NT-proBNP Median (Q1, Q3) (pg/ml)	*p*-value
Troponin		
Positive	544 (-)	0.005
Negative	140 (97, 329)	
Pulmonary Edema		
Present	544 (-)	
Absent	141 (99, 351)	
ECG Findings		
Normal	134.5 (96.25, 288.25)	0.001
ST changes	544 (-)	
T inversion	484 (-)	
Pathologic Q wave	527 (-)	
Overall CV complications		
Present	514 (411.75, 725.5)	< 0.001
Absent	134.5 (96.25, 288.25)	

A ROC curve was constructed to predict postoperative cardiovascular complications using preoperative NT-proBNP levels. A 332.5 pg/ml cut-off value was identified as the optimal predictor of postoperative cardiovascular complications, representing the optimal tradeoff between sensitivity and specificity. The area under the curve (AUC) was 0.924 (95% confidence interval [CI] 0.85 to 0.99, *p* = 0.001), yielding a sensitivity of 100%, specificity of 79.2%, PPV of 40%, and NPV of 100% (Fig. 3). A logistic regression was performed, and there was no significant correlation between age or gender and postoperative cardiovascular complications (*p* = 0.4, *p* = 0.7, respectively).

**Fig. 3:** ROC curve for preoperative NT-proBNP level and prediction of postoperative cardiovascular complications

## Discussion

Determining the risk of postoperative cardiovascular complications in patients undergoing noncardiac surgery (NCS) is fundamental to every preoperative assessment. Reduced postoperative cardiovascular complications after NCS in recent years may be partly due to better risk assessment. Several approaches have been proposed to increase the efficacy of these measures, yield more accurate results, and improve the cost/benefit of the process.

In this study, we sought to compare the efficiency of measuring NT-proBNP level as a cardiac biomarker and MPS as a non-invasive stress imaging tool in predicting postoperative cardiovascular complications before performing NCS. Our results have revealed that NT-proBNP and MPS are perfectly sensitive in identifying at-risk patients. However, using the cut-off value of 332.5 pg/ml for the NT-proBNP level resulted in roughly 13% more specificity and 20% more positive predictive value in detecting high-risk patients than the MPS.

Several studies have investigated the mechanisms underpinning perioperative myocardial infarction. On top of these mechanisms is increased myocardial oxygen demand and concurrent inadequate supply due to high-grade coronary stenosis, which accounts for 55% of cases [11]. Another proposed explanation is plaque rupture and subsequent coronary obstruction secondary to surgical stress, which comprises 26% of patients [11]. Yet studies have shown that a large proportion of the latter mechanism occurs in the setting of mild stenosis on preoperative assessments [12].

Stress imaging techniques, such as MPS, mainly fail to detect a mild obstruction and subclinical plaque formation as a significant factor predisposing patients to thrombotic events [13]. Furthermore, MPS's incremental predictive value is limited to high- or moderate-risk surgeries and cannot be implemented in low-risk settings [14]. The low positive predictive value of the technique also questions the rationale behind its utilization, except for particular indications [8, 15]. A 2019 meta-analysis also explains that there is no evidence of the effectiveness of preoperative stress imaging in perioperative mortality reduction [16].

In recent years, the application of cardiac biomarkers in preoperative cardiovascular assessment, especially NT-proBNP, has expanded, evident in the latest guidelines on this issue [17]. Although the 2022 European Society of Cardiology (ESC) guideline has recommended that NT-proBNP levels higher than 125 pg/ml be considered abnormal [6], there is no consensus among studies to this date on the optimal cut-off value to recognize high-risk patients before NCS. This variance may be due to renal function, age, and body mass index (BMI), which influence the NT-proBNP level and differ among studies [17]. Renal dysfunction and reduced glomerular filtration rate (GFR) lead to lower NT-proBNP excretion and elevated serum level. Thus, its prognostic value is unimportant in GFR lesser than 30 ml/min/1.73 m^2^ [18]. The NT-proBNP level also is inversely associated with BMI and values lower in obese patients [19]. These factors and age-specific cut-offs for NT-proBNP [20] should be considered when interpreting the association between this biomarker and postoperative cardiovascular complications.

Given the aforementioned shortcomings of MPS and the higher predictive value of NT-proBNP testing, our study suggests utilizing preoperative NT-proBNP assessment as a more specific substitute for MPS in patients undergoing high- to moderate-risk elective NCS with poor functional capacity and high clinical risk or likelihood of CAD. Compared to an MPS, this approach averts unnecessary delay before surgery, reduces the expenses, and offers a higher level of accessibility and feasibility, as well as a more specific prediction of postoperative cardiovascular complications with high diagnostic sensitivity. Nevertheless, whether interventions based on NT-proBNP level would translate into a reduction in postoperative cardiovascular morbidity and mortality is yet to be investigated.

### Limitations

This study encompasses several limitations. Our study population was relatively small, hampering its results from being generalizable to a larger population. We also did not have access to patients’ baseline comorbidities and characteristic cardiac risk factors and the data were only stored as their calculated RCRI score. Due to our limited cases, further analysis of patients' factors affecting NT-proBNP levels, such as GFR, age, and BMI, could not yield reliable outcomes. As the MPS result in our study was a categorical variable, it was impossible to draw a ROC curve and define a cutoff for it. Hence, it was not feasible to provide a direct comparison between MPS and NT-proBNP accuracy. Additionally, further follow-up of patients is warranted to discover the power of this approach in predicting mid and long-term postoperative cardiovascular complications.

## Conclusion

Our results suggest an extended application of preoperative NT-proBNP level assessment to evaluate the incidence of postoperative cardiovascular complications and take proper measures before and during surgery to reduce these complications. This study reveals the additive specificity of NT-proBNP over MPS as a stress imaging technique (Fig. 4). This approach can spare the extra expense and time imposed by MPS and reduce false positive results.

**Fig. 4:** Summary of the study results

## Data Availability

All data generated or analyzed during this study are available from the corresponding author upon request.

## Abbreviations

MPS: Myocardial perfusion scan
NT-proBNP: N-terminal pro-b-type natriuretic peptide
PPV: Positive predictive value
NPV: Negative predictive value
